# Pain Treatment Evaluation in COVID-19 Patients with Hesitant Fuzzy Linguistic Multicriteria Decision-Making

**DOI:** 10.1155/2021/8831114

**Published:** 2021-02-01

**Authors:** G. Didem Batur Sir, Ender Sir

**Affiliations:** ^1^Department of Industrial Engineering, Gazi University, Ankara 06570, Turkey; ^2^Department of Algology and Pain Medicine, Health Sciences University, Gülhane Training and Research Hospital, Ankara 06010, Turkey

## Abstract

The coronavirus disease 2019 (COVID-19) has emerged as a worldwide pandemic since March 2020. Although most patients complain of moderate or severe pain, these symptoms are generally underestimated and appropriate treatment is not applied. This study aims to guide physicians in selecting and ranking various alternatives for the treatment of pain in COVID-19 patients. However, the choice of treatment for pain requires the consideration of many different conflicting criteria. Therefore, we have studied this problem as a multicriteria decision-making problem. Throughout the solution procedure, first, the criteria and subcriteria affecting the preferences are defined. Then, weight values are determined with respect to these criteria, as they have different degrees of importance for the problem. At this stage, hesitant fuzzy linguistic term sets (HFLTSs) are used, and thus, experts can convey their ideas more accurately. In this first phase of the study, an HFLTS integrated Analytic Hierarchy Process (AHP) method is utilized. Subsequently, possible treatment alternatives are evaluated by using the Vise Kriterijumska Optimizacija I Kompromisno Resenje (VIKOR) method. According to the results obtained by considering expert evaluations, the most preferred treatment is the administration of paracetamol, followed by interventional treatments, opioids, and nonsteroidal anti-inflammatory drugs (NSAIDs), respectively. With this study, it is ensured that a more accurate method is followed by eliminating possible mistakes due to the subjective evaluations of experts in the process of determining pain treatment. This method can also be used in different patient and disease groups.

## 1. Introduction

The coronavirus disease 2019 (COVID-19), a highly contagious virus disease, was first found in China in December 2019. The World Health Organization (WHO) declared COVID-19 as a pandemic in March 2020. To date, more than forty million patients and approximately twelve hundred thousand deaths have been reported worldwide [1]. Fever, cough, breathlessness, malaise, diarrhea, anosmia, and pain complaints are the most common symptoms in COVID-19. Although standard protocols and treatment algorithms have not yet been established for the treatment of the disease, antiviral treatments are prioritized, and serious complications such as acute respiratory distress syndrome (ARDS) are considered primarily. However, this approach has caused the pain complaints of patients to often be ignored. Therefore, the choice of pain treatment modality in COVID-19 patients is still a crucial problem. No consensus has yet been reached on this issue. The treatments for these pain complaints often differ according to the personal experiences and preferences of the practitioners.

Multicriteria decision-making (MCDM) analysis was introduced to healthcare as an appropriate decision support framework for solving complex problems using accessible approaches [2]. The nature of decisions relevant in healthcare systems, which require multiple criteria to be considered simultaneously, is the basis of several studies conducted in this domain as well as future studies. Focusing on the current MCDM studies, many studies focusing on the treatment options for different diseases have been conducted. Having a closer look on the examples done in recent years, Suner et al. [3] developed a decision support tool for physicians in order to select the most beneficial rectal cancer treatment using the Analytic Hierarchy Process (AHP) together with the decision trees. Lopez and Gunasekaran [4] evaluated H1N1 influenza vaccination strategies using fuzzy logic-based Vise Kriterijumska Optimizacija I Kompromisno Resenje (VIKOR) method. Hsu et al. [5] used AHP in order to assess the choice of oral phosphodiesterase type 5 inhibitors for the treatment of erectile dysfunction. Balubaid and Basheikh [6] tried to select the appropriate oral hypoglycemic agent for use among newly diagnosed patients with type 2 diabetes. Hancerliogullari et al. [7] evaluated anesthesia methods for circumcision surgery by using fuzzy AHP and fuzzy TOPSIS. Ji et al. [8] applied a fuzzy decision-making-based approach for the treatment selection problem of a particular patient with verruca plantaris. Malekpoor et al. [9] presented a TOPSIS and case-based reasoning method to prescribe a suitable dose plan for prostate cancer. Eghbali-Zarch et al. [10] dealt with the problem of pharmacological therapy selection of type 2 diabetes and proposed a computer-aided medical decision support tool using a fuzzy MCDM model including fuzzy Multi-Objective Optimization by a Ratio Analysis plus the Full Multiplicative Form (MULTIMOORA) and fuzzy Stepwise Weight Assessment Ratio Analysis (SWARA). Sir and Batur Sir [11] evaluated nonpharmacological treatment options for patients with chronic cancer pain by an MCDM procedure. Samanlioglu [12] tried to determine the best intervention strategies for influenza using fuzzy AHP and fuzzy VIKOR. Besides, there are some recent studies on decision-making [13] and optimization [14] within the focus on COVID-19 disease.

In this study, the selection and ranking of different treatment options were investigated in patients with mild to moderately severe COVID-19. Hence, effective criteria were determined primarily in consideration of existing relevant literature and the opinions of physicians from different specialties. These criteria were then weighted according to their relative importance with respect to each other. Finally, the most commonly used and appropriate treatments were determined and analyzed according to these criteria, assigning higher importance to those with higher weights.

At this point, another issue needs to be addressed. In classical MCDM studies, it is accepted that all evaluation data are known precisely. However, the ambiguities in human preferences and the possibility of confrontation with the situations of decision-makers make this assumption invalid. Fuzzy logic and fuzzy sets are being used to handle such vague and imprecise information. Various extensions have been developed for situations where ordinary fuzzy logic is insufficient. For example, interval value type 2 fuzzy sets, which are a special case of type 2 fuzzy sets, are claimed to provide low computational complexity and high flexibility to decision-makers focusing on MCDM problems [15].

Although all these definitions have been shown to be used effectively in various problems, they are still limited to situations where decision-makers are expected to determine a single value. Hesitant fuzzy sets have arisen as another extension that try to manage situations where a set of values are possible in the definition process of the membership of an element [16]. In multicriteria problems where the levels of importance of the decision criteria are different from each other, the hesitation of decision-makers may cause significant changes in the final solution. In such cases, the use of hesitant fuzzy linguistic term set (HFLTS) has been introduced recently and is a frequently used method. The use of hesitant fuzzy assessments enables the judgments of decision-makers to be more reliable and informative regarding the decision-making process [17]. Zhang et al. [18], Liang et al. [19], Dong et al. [20], Li et al. [21], Wu et al. [22], Sun et al. [23], Zheng et al. [24], Wu et al. [25], Xiao et al. [26], Wu et al. [27], and Wu et al. [28] are some of the most recent studies.

The generalized framework created by Watróbski et al. [29] was used to determine the solution method to be used in the study. In the problem that we deal with, criteria with different weights were taken into consideration and the alternatives were evaluated on a quantitative scale. Within the framework of the rules for determining the most suitable MCDM method presented by Watróbski et al. [29], the most appropriate method to be used for the ranking and selection problem in such problems was determined to be AHP + VIKOR. Besides, taking into account the hesitant nature of the decision-makers mentioned earlier, the HFLTS concept was also used. Thus, it is concluded that the HFLTS integrated AHP method was used in the first stage, where the criteria weights were determined, and the VIKOR method was appropriate in the second stage, where the alternatives were evaluated.

The main motivation for this study is to guide physicians in selecting and ranking alternatives that can be used to treat the pain symptoms observed in COVID-19 patients. For this purpose, an HFLTS integrated AHP + VIKOR methodology is proposed within the context of MCDM.

This paper is organized as follows. The next section presents the problem-specific treatment alternatives and evaluation criteria, together with the steps of calculating the weight values, and the related ranking and selection methodology. In the Results and Discussion section, we focus on real data with respect to the evaluations of experts and present the final results. Finally, concluding remarks and future directions are presented.

## 2. Materials and Methods

### 2.1. Treatment Alternatives

In this study, the objective was to evaluate the most appropriate pain treatment in mild to moderate COVID-19 patients. The considered treatment alternatives were paracetamol (Alternative 1), nonsteroidal anti-inflammatory drugs (NSAIDs) (Alt. 2), opioids (Alt. 3), and interventional procedures (Alt. 4). In determining these treatments, a group of evaluators consisting of a pain physician, an anesthesiologist, a pulmonologist, an internal medicine physician, and an infectious diseases physician were consulted. A literature review was also conducted.

Paracetamol (acetaminophen) is the most commonly used medication to treat fever and pain in both Europe and the United States [30]. It is considered to not affect the immune system because it has minor anti-inflammatory effects. It is generally used for mild to moderate pain or can be used for stronger pain by combining NSAIDs and opioids. As it is metabolized in the liver, its effect on kidney function is minimal and does not cause gastric problems.

Along with fever, NSAIDs are often used to treat acute or chronic inflammatory pain conditions. NSAIDs act by inhibiting cyclooxygenase enzymes (COX-1 or COX-2). They are divided into two groups, namely, nonselective and COX-2-selective. The COX-2-selective NSAIDs are more reliable than the nonselective group in terms of the risk of stomach ulcers and bleeding. NSAIDs should be used cautiously in patients with uncontrolled hypertension, coronary diseases, kidney disease, and stomach problems. Although there are contradictory statements about ibuprofen, which is an NSAID, there is no strong evidence to suggest that the use of NSAIDs adversely affects the disease [31].

Opioids act on the nervous system and block pain communication between the brain and the body. They are often used in the management of moderate-to-severe pain. Unlike paracetamol and NSAIDs, they are not used to treat fever or inflammation. However, they have some advantages over other pain relievers. They have anxiolytic effects, such that they suppress fear and anxiety in patients. Additionally, cough and diarrhea are common symptoms in COVID-19 patients, and opioids, especially codeine, have antitussive and antidiarrheal effects. However, opioids have some undesirable side effects, including respiratory depression and addiction. Therefore, opioids should not be preferred for treating COVID-19 patients with respiratory failure symptoms. In addition, to prevent addiction, opioids used in the disease treatment should be reduced gradually and discontinued in the following recovery period.

In cases that are resistant to drug treatments or in patients with drug-related side effects, interventional pain treatment is another alternative. In severe neuralgias and headaches, the greater occipital nerve block, supraorbital, and mental nerve block can be applied. Procedures such as the transnasal sphenopalatine block that may cause aerosol formation should be avoided. Furthermore, local anesthetic injections can be applied to the painful regions in severe lower-back, neck, and muscle aches. In such patients experiencing severe pain, corticosteroid injections should not be preferred due to their immunosuppressive effects.

### 2.2. Evaluation Criteria

Establishing the problem hierarchy by determining the criteria affecting the ranking of appropriate treatments is one of the main objectives of this study. The problem hierarchy shows the evaluation criteria for this purpose, together with the goal discussed in the problem. Similar to the process of determining the alternatives, the literature on the choice of treatment was researched, and the opinions of the experts were used while defining the criteria. As a result, it is determined that the evaluation should be conducted by considering the pain characteristics (C1), coexisting symptoms (C2), comorbid diseases (C3), mood dysregulation (C4), and possible risks (C6). The hierarchical structure created, including the relevant subcriteria, is presented in Figure 1.

As can be seen from the figure, the first main criterion is pain characteristics, and its subcriteria are pain region (C11), pain intensity (C12), and pain duration (C13). The region of the pain is either localized or the whole body. In patients, pain may occur only in a single area such as head, abdomen, or waist, or sometimes it can be seen as whole body pain. It would be beneficial to prefer the treatments targeting the pain area. Pain intensity can be classified as mild-moderate or severe. Pain duration can be classified as intermittent/short-term pain and continuous pain. It is appropriate to give medicines in the form of infusions in continuous pain or to give drugs with long duration of action at regular intervals. In short-term and intermittent pain, short-acting analgesics should only be given as needed.

The second main criterion is the coexisting symptoms and its subgroups are fever (C21), diarrhea (C22), and cough (C23). Fever can also accompany malaise and sometimes whole body pain. Cough is one of the most common symptoms of COVID-19 and often causes chest pain. In diarrhea, abdominal pain is a common form of pain. In cases of cough and diarrhea, treatments having antitussive and antidiarrheal effects are preferable.

The third main criterion is that comorbid diseases exist. Subcriteria are chronic obstructive pulmonary disease (COPD) (C31), kidney dysfunction (C32), and stomach problems (C33) such as peptic ulcer and gastritis. For example, in cases with COPD, there is a predisposition to respiratory depression that should be taken into consideration.

The fourth main criterion is mood dysregulation. Subcriteria are anxiety (C41) and depression (C42). In most diseases, the mood of patients is impaired. Moreover, in diseases such as COVID-19 that require high rates of hospitalization, patients' fear of death is a serious source of anxiety. Depression is inevitable in cases with prolonged hospitalization or when the treatment process is negative. In these patients, early treatment of anxiety will reduce the risk of developing problems such as depression, panic attack, and posttraumatic stress disorder in the postdisease period.

Subcriteria of possible risks, which is our last main criterion, are as follow-up risk (C51), complication risk (C52), and addiction risk (C53). The risk of follow-up is related to situations where the patient should be closely monitored from a medical point of view. In patients at risk of follow-up, the risk of complications, the second subcriterion, also increases. For such cases, less risky treatments can be preferred. It is important not to prefer drugs with addictive potential as a priority and to avoid prolonged exposure if used.

### 2.3. Weighting of the Criteria

At the next stage, the criteria weights that will indicate the importance of the mentioned criteria and subcriteria in terms of the selection and ranking problem should be determined. The use of the AHP, which is frequently preferred in the literature in determining the criteria weights, is decided to be appropriate at this stage. AHP is one of the MCDM techniques developed by Saaty in 1977 [32]. It is a mathematical method that takes into account the priorities of the group or individuals and evaluates the qualitative and quantitative variables together [33].

As it is mentioned before, one of the most important problems that we encounter in the stages where expert evaluations are needed is the hesitations that decision-makers experience. HFLTS is used to prevent such hesitations and to facilitate the evaluations of the consulted experts. The approach was originally proposed by Rodríguez et al. [16]. In this stage, the main steps of the HFLTS-based AHP methodology defined by Tüysüz and Şimşek [34] are used. Assuming *S*={*s*_0_,…, *s*_*g*_} is a linguistic term set, the elements of the context-free grammar *G*_*H*_={*V*_*N*_, *V*_*T*_, *I*, *P*} are defined as follows:

(1) $$\begin{array}{c} V_{N}=\left\{\langle \text{primary term}\rangle ,\langle \text{composite term}\rangle ,\langle \text{unary relation}\rangle ,\langle \text{binary relation}\rangle ,\langle \text{conjunction}\rangle \right\},\\ V_{T}=\left\{\text{lower than},\text{greater than},\text{between},\text{at least},\text{at most},\text{and},s_{0},s_{1},\ldots ,s_{g}\right\},\\ I\in V_{N},\\ P=\left\{\begin{array}{c} I⩴\langle \text{primary term}\rangle |\langle \text{composite term}\rangle ,\\ \langle \text{composite term}\rangle ⩴\langle \text{unary relation}\rangle \langle \text{primary term}\rangle \;|\\ \langle \text{binary relation}\rangle \langle \text{primary term}\rangle \langle \text{conjunction}\rangle \langle \text{primary term}\rangle ,\\ \langle \text{primary term}\rangle ≔=s_{0}\left|s_{1}\right|,\ldots ,|s_{g},\\ \langle \text{unary relation}\rangle ⩴\text{lower than }\left|\text{greater than}\right|\text{at least}|\text{at most},\\ \langle \text{binary relation}\rangle ⩴\text{between},\langle \text{conjunction}\rangle ⩴\text{and} \end{array}\right\}. \end{array}$$

Assuming that *E*_*G*_*H*__ is a function that converts expressions into HFLTS, the following transformations are used for this purpose [16]:

(2) $$\begin{array}{c} E_{G_{H}}\left(s_{i}\right)=\left\{s_{i}|S_{i}\in S\right\},\\ E_{G_{H}}\left(\text{at most }s_{i}\right)=\left\{s_{j}|s_{j}\in S\text{ and }s_{j}\leq s_{i}\right\},\\ E_{G_{H}}\left(\text{lower than }s_{i}\right)=\left\{s_{j}|s_{j}\in S\text{ and }s_{j}<s_{i}\right\},\\ E_{G_{H}}\left(\text{at least }s_{i}\right)=\left\{s_{j}|s_{j}\in S\text{ and }s_{j}\geq s_{i}\right\},\\ E_{G_{H}}\left(\text{greater than }s_{i}\right)=\left\{s_{j}|s_{j}\in S\text{ and }s_{j}>s_{i}\right\},\\ E_{G_{H}}\left(\text{between }s_{i}\text{ and }s_{j}\right)=\left\{s_{k}|s_{k}\in S\text{ and }s_{i}\leq s_{k}\leq s_{j}\right\}. \end{array}$$

The envelope of an HFLTS, env(*H*_*S*_), is a linguistic interval whose limits are obtained by its maximum value and minimum value:

(3) $$\begin{array}{c} \text{env}\left(H_{S}\right)=\left[H_{S^{-}},H_{S^{+}}\right],\;H_{S^{-}}\leq H_{S^{+}}, \end{array}$$

where *H*_*S*^−^_=min(*s*_*i*_)=*s*_*j*_, *s*_*i*_ ∈ *H*_*S*_ and *s*_*i*_ ≥ *s*_*j*_, ∀*i* and *H*_*S*^+^_=max(*s*_*i*_)=*s*_*j*_, *s*_*i*_ ∈ *H*_*S*_ and *s*_*i*_ ≤ *s*_*j*_, ∀*i*.

The main steps of the algorithm are defined as follows [34]:

Step 1: define the semantics and syntax of the linguistic term set *S* and the context-free grammar *G*_*H*_.
Step 2: gather the pairwise comparisons from the experts. In the domain of group decision-making, *m* decision-makers (*E*={*e*_1_, *e*_2_,…, *e*_*m*_}) try to select the best alternative among *n* alternatives (*X*={*x*_1_, *x*_2_,…, *x*_*n*_}), where *m* > 1 and *n* > 1. In this case, a matrix composed of preference relations (*p*^*k*^*s*) is formed as in the following equation:
  (4) $$\begin{array}{c} p^{k}=\left(\begin{array}{ccc} p_{11}^{k} & \cdots & p_{1m}^{k}\\ \vdots & \ddots & \vdots \\ p_{n1}^{k} & \cdots & p_{nm}^{k} \end{array}\right), \end{array}$$
where *p*_*ij*_^*k*^ shows the degree of preference of the alternative *x*_*i*_ over *x*_*j*_ according to expert *e*_*k*_.
Step 3: transform the preference relations into HFLTS by using the transformation function *E*_*G*_*H*__. For each HFLTS, obtain an envelope [*p*_*ij*_^*k*−^, *p*_*ij*_^*k*+^].
Step 4: obtain the pessimistic and optimistic collective preference relations (*P*_*C*_^−^ and *P*_*C*_^+^). Compute the pessimistic and optimistic collective preference for each alternative using 2-tuple sets. The 2-tuple set associated with *S* is defined as *S*=*Sx*[0.5, 0.5). The function Δ : [0, *g*]⟶*S* is given as
  (5) $$\begin{array}{c} \Delta \left(\beta \right)=\left(s_{i},\alpha \right)\text{ with }\left\{\begin{array}{c} i=\text{round}\left(\beta \right),\\ \alpha =\beta -i, \end{array}\right. \end{array}$$
where round assigns to *β* the integer number *i* ∈ {0,1,…, *g*} closest to *β* and Δ^−1^ : *S*⟶[0, *g*] is defined as in the following equation:
  (6) $$\begin{array}{c} \Delta^{-1}\left(s_{i},\alpha \right)=i+\alpha . \end{array}$$
Step 5: build a vector of intervals *V*^*R*^=(*p*_1_^*R*^, *p*_2_^*R*^,…, *p*_*n*_^*R*^) of collective preferences for the alternatives *p*_*i*_^*R*^=[*p*_*i*_^−^, *p*_*i*_^+^].
Step 6: calculate the midpoints of the intervals and normalize the results in order to find the weights.

### 2.4. Ranking and Selection of the Alternatives

After the criterion weights are determined, the alternatives are evaluated based on these criteria. For this purpose, VIKOR method is used in this study. The VIKOR method, which was first referred to by Opricovic [35], was used in 2004 by Opricovic and Tzeng [36] in the solution of MCDM problems. The meaning of VIKOR, which is the abbreviation of Vise Kriterijumska Optimizacija I Kompromisno Resenje, is multicriteria optimization and compromised solution. The basis of the method is the creation of a compromise solution within the framework of alternatives and the evaluation criteria. This compromised solution is the closest solution to the ideal solution [37]. In the method, by creating a multicriteria ranking index for alternatives, it is possible to make the decision closest to the ideal solution under certain conditions. The comparative order is achieved by comparing the measure of closeness to the ideal alternative [38].

The steps of the method can be summarized as follows:

Step 1: the best (*f*_*i*_^*∗*^) and worst (*f*_*i*_^−^) values are determined for each of the evaluation criteria. If criterion *i* (for *i*=1,2,…, *n*) is defined in terms of “benefit” for evaluation, *f*_*i*_^*∗*^ and *f*_*i*_^−^ can be expressed as follows:
  (7) $$\begin{array}{c} f_{i}^{*}=\underset{j}{\max}f_{ij},\\ f_{i}^{-}=\underset{j}{\min}f_{ij}, \end{array}$$
where *f*_*ij*_ represents the value of *i*^th^ criterion for the *j*^th^ alternative. Throughout the solution procedure of this study, binary values are determined for *f*_*ij*_'s.
Step 2: *S*_*j*_ and *R*_*j*_ values are calculated for each evaluation unit. *w*_*i*_ represents the criteria weights.
  (8) $$\begin{array}{c} S_{j}=\frac{\sum_{i=1}^{n}w_{i}\left(f_{i}^{*}-f_{ij}\right)}{\left(f_{i}^{*}-f_{i}^{-}\right)},\\ R_{j}=\max\left[\frac{w_{i}\left(f_{i}^{*}-f_{ij}\right)}{\left(f_{i}^{*}-f_{i}^{-}\right)}\right]. \end{array}$$
Step 3: *Q*_*j*_ values are calculated for each evaluation unit.
  (9) $$\begin{array}{c} Q_{j}=\frac{v\left(S_{j}-S^{*}\right)}{\left(S^{-}-S^{*}\right)}+\frac{\left(1-v\right)\left(R_{j}-R^{*}\right)}{\left(R^{-}-R^{*}\right)}. \end{array}$$
In equation (6), *S*^*∗*^=min_*j*_*S*_*j*_, *S*^−^=max_*j*_*S*_*j*_, *R*^*∗*^=min_*j*_*R*_*j*_, and *R*^−^=max_*j*_*R*_*j*_. The value of *v* indicates the weights of the majority of the criteria, in other words, the maximum group benefit. While the value of *v* represents the weight for the strategy that provides the maximum group benefit, the value of (1 − *v*) indicates the weight of the minimum regret of the opponents [38]. Usually, *v*=0.5 is used [39].
Step 4: calculated values of *Q*_*j*_, *S*_*j*_,  and *R*_*j*_ are listed. The evaluation unit with the smallest *Q*_*j*_ value is expressed as the best option in the alternative group.
Step 5: two conditions must be met in order for the obtained result to be considered valid. Only in this way can an alternative with the minimum *Q* value be considered the best or the most suitable.

**Condition 1 (acceptable advantage).**

It states that there is a distinct difference between the best and the closest to the best options:

(10) $$\begin{array}{c} Q\left(P_{2}\right)-Q\left(P_{1}\right)\geq D\left(Q\right). \end{array}$$

In this equation, *P*_1_ is the first best alternative with the lowest *Q* value and *P*_2_ is the second best alternative. It is expressed as follows: (*Q*)=1/(*j* − 1). *j* indicates the number of evaluation units. If the number of evaluation units is less than 4, then *D*(*Q*)=0.25 [40].

**Condition 2 (acceptable stability).**

Alternative *P*_1_ with the best *Q* value should have achieved the best score in at least one of the *S* and *R* values.

If one of the two specified conditions cannot be met, the compromised solution set is recommended consisting of

- *P*_1_ and *P*_2_, alternatives If Condition 2 is not met
- *P*_1_, *P*_2_,…, *P*_*M*_ alternatives which are expressed by considering the inequality of *Q*(*P*_*M*_) − *Q*(*P*_1_) ≥ *D*(*Q*) If Condition 1 is not met, [36]

## 3. Results and Discussion

The method described in the previous section was applied to the problem of pain treatment ranking and selection in mild to moderate COVID-19 patients. As mentioned before and presented in Figure 1, the criteria that are effective in the problem under consideration were determined under five main titles and a total of 14 subtitles. In order to determine the relative weights of these criteria, the following semantics and syntax of the linguistic term set *S* was defined:

(11) $$\begin{array}{c} S=\left\{\begin{array}{c} \begin{array}{c} \text{absolutely low}\left(\text{n}\right),\\ \text{very low}\left(\text{vl}\right),\\ \text{low}\left(\text{l}\right), \end{array}\\ \text{medium}\left(\text{m}\right),\\ \text{high}\left(\text{h}\right),\\ \text{very high}\left(\text{vh}\right),\\ \text{absolutely high}\left(\text{ah}\right) \end{array}\right\}. \end{array}$$

At this stage of the study, the calculations performed on the basis of the main criteria were given so that the reader would have a better insight over the method steps. First, pairwise evaluations were asked from the experts presenting their linguistic comparisons related to the main criteria. These evaluations are given in Table 1. They were then converted to envelops for each of the HFLTSs. Obtained envelops are presented in Table 2. Using the scale given in Table 3, the pessimistic and optimistic collective preferences were determined, which are given in Table 4.

At the last step, after converting the linguistic intervals into interval utilities, the midpoints of these utilizes were calculated and normalized in order to obtain the weights. Related interval values and midpoints, together with the weights obtained for the main criteria, are given in Table 5. According to these values, when we list the main criteria, the most important parameter in the selection and ranking of treatment is comorbid diseases. These ones both cause the disease to be severe and affect the choice of treatment. The second main criterion is the possible risks. It should be aimed to relieve the pain of patients by avoiding the risks as much as possible. Other main criteria are coexisting symptoms, pain characteristics, and mood dysregulation, respectively. All of these criteria are important and may differ from person to person. However, it would be appropriate to take this ranking into consideration while establishing a treatment protocol.

Applying the same procedure for both the main and subcriteria, the resulting weights given in Table 6 were obtained. When the subcriteria were examined separately, it was found that the most important criterion was the presence of COPD. In COVID-19 patients, respiratory distress is often encountered when the disease progresses. Furthermore, COPD itself can lead to the development of respiratory distress or a more severe course of the disease. The second subcriterion found was the risk of complications. During pain management, there may be many complications such as respiratory depression, kidney failure, stomach bleeding, and drug reactions. It is important to determine the risks of these complications in advance and to prefer the lowest-risk treatment. The third criterion was fever. High fever often causes malaise and pain in patients. Kidney dysfunction took the fourth place. In such patients who are currently unable to use most drugs, treatment should be determined accordingly. It was determined that the next important subcriterion was the presence of anxiety. If anxiety is not treated early, patients may develop conditions such as depression and stress disorder in the chronic period. Also, generalized anxiety disorder reduces patients' compliance to treatment. Other subcriteria in order of importance were cough, risk of addiction, stomach problems, pain region, pain severity, follow-up risk, diarrhea, depression, and duration of pain, respectively.

After defining the criteria and subcriteria, quantitative assessment values were assigned for possible situations, and alternative treatments were scored. As it is previously defined, *f*_*ij*_ represents the value of *i*^th^ criterion for the *j*^th^ alternative and is a binary value. Values of *f*_*ij*_'s here are determined according to the convenience of the alternative for the existence of that specific criterion. For example, under the subcriterion C11, alternatives Alt. 1, Alt. 2, and Alt. 3 are preferred for whole body pain, whereas alternative Alt. 4 is not appropriate for this indication. All other values were assigned accordingly. Once the alternatives are scored, related best (*f*_*i*_^*∗*^) and worst (*f*_*i*_^−^) values are determined for each criterion. At this point, while defining *f*_*i*_^*∗*^ and *f*_*i*_^−^, 1 and 0 values were assigned for the best and worst values, respectively, with the aim of choosing the most effective treatment alternative with respect to each criterion. The values obtained as a result of this scoring are given in Table 7.

Then, *S*_*j*_ and *R*_*j*_ values were calculated taking the previously calculated weight (*w*_*i*_) values into account. At the next step, *S*^*∗*^, *S*^−^, *R*^*∗*^, and *R*^−^ were defined, and *Q*_*j*_ was obtained using equation (9). Calculated values of *S*_*j*_, *R*_*j*_, *Q*_*j*_ and related rankings are given in Table 8.

Alternative 1, namely, paracetamol, is the best ranked treatment method based on the *Q*_*j*_ values. Checking the two conditions of the method, we see that this alternative has both acceptable and stability advantages over the other alternatives. Among the others, Alt. 4 (interventional procedures), Alt. 3 (opioids), and Alt. 2 (NSAIDs) seem to be the second, third, and fourth treatment methods, respectively. However, they do not have a comparative advantage over each other, so we conclude that they all are the second ranked alternative treatments for these patients having slight changes of “costs” and “benefits.”

### 3.1. Discussion

COVID-19 patients frequently have pain complaints in different forms. However, in these patients, pain-relieving treatments are often ignored and even avoided due to the current uncertainties about the disease and the published confusing reports. Despite the high prevalence of pain in these patients, there is no concrete guide on pain management, and the choice of treatment is based on personal decisions and preferences. In such cases, there are many independent and often contradictory criteria, and all these criteria should be considered for making the decision. In this study, considering the complex structure of the problem of determining the appropriate treatment method for COVID-19 patients with pain complaints, we attempted to use a scientific approach.

In this study, the evaluations of specialists and the related literature were considered. In particular, the evaluations made by the experts were of great importance in determining the criteria and their relative weights while comparing alternatives. Regarding this situation, HFLTS definitions were utilized by predicting the hesitations of experts in the decision-making role. Thus, decision-makers were able to make subjective evaluations more easily, and the validity and reliability of their assessments improved. Furthermore, by rigorously reviewing the MCDM literature, it was found that the AHP + VIKOR approach is the most suitable method for this specific decision problem. Consequently, the method that we have applied is determined to be an HFLTS integrated AHP + VIKOR procedure. As a result of our analysis, the most preferable treatment was determined to be paracetamol, followed by interventional treatments, opioids, and finally NSAIDs.

Paracetamol is a drug that has both antipyretic and analgesic effects. It is also safe in terms of side effects. It has no contraindications, except for severe liver failure. It can also be synergistically combined with other analgesic drugs. As a result, paracetamol is determined to be the first choice in the treatment of pain in COVID-19 patients. Interventional pain treatments are in second place. Some of the reasons include the procedure being targeted to the painful area instead of the whole body, lack of systemic side effects, and low risks of follow-up and complications. Despite the risk of respiratory depression in the acute period and addiction in the long term, the third ranked method of treatment is opioids. Its main advantages are use in severe pain levels and positive effects on coexisting symptoms such as cough and diarrhea. Additionally, it can be used in patients with kidney dysfunction and stomach problems. The most important reason for NSAIDs to be least preferred is the occurrence of systemic side effects and the risks of gastric and nephrological complications. In addition, negative reports about NSAIDs have also negatively affected the preference of physicians for these drugs.

## 4. Conclusions

The main contribution of this study is to provide a guideline regarding pain management in COVID-19 patients and to determine the most appropriate treatment modality for these cases. The HFLTS integrated AHP + VIKOR procedure is proposed for this purpose. Accordingly, it is predicted that paracetamol should be used first in these patients, and then interventional methods, opioids, and NSAIDs are preferred. As previously mentioned, this is the first such study and the results obtained here are expected to guide physicians in treatment planning. This approach can also be used to address other decision-making problems in healthcare management.

The most evident advantage of the proposed method is the use of HFLTS definitions. Through these definitions, decision-makers can make subjective evaluations more easily, and the validity and reliability of their assessments are improved. Second, the problem of determining the appropriate treatment method for COVID-19 patients with pain complaints has a complex structure and necessitates the use of a scientific approach. This study presents this scientific approach in the context of the relevant MCDM literature.

This study has specific limitations, such as the number of experts consulted. Increasing this number can possibly reduce bias related to the subjective evaluations of decision-makers. The second limitation is the exclusion of the age factor, which affects both the progress of the disease and the metabolism of the drugs in patients. In addition, newly proposed methods may be used in future studies. Some examples include recent extensions on HFLTSs, such as probabilistic hesitant fuzzy sets [41–43] and double-hierarchy HFLTSs [44]. By solving the problem through these methods, a comparison can be made with the current approach.

## Figures and Tables

**Figure 1:** Hierarchical organization of the decision-making criteria.

**Table 1:** Pairwise evaluations of the main criteria.

	C1	C2	C3	C4	C5
*Pain physician*					
C1	—	Between (l and m)	Between (vl and l)	Between (h and vh)	Between (m and h)
C2	Between (m and h)	—	Between (l and m)	Is (vh)	Between (h and vh)
C3	Between (h and vh)	Between (m and h)	—	At least (vh)	Is (vh)
C4	Between (vl and l)	Is (vl)	At most (vl)	—	Between (l and m)
C5	Between (l and m)	Between (vl and l)	Is (vl)	Between (m and h)	—

*Anesthesiologist*					
C1	—	Between (l and m)	At most (l)	Is (m)	Between (vl and l)
C2	Between (m and h)	—	Between (vl and l)	Between (h and vh)	Between (l and m)
C3	At least (h)	Between (h and vh)	—	At least (vh)	Between (m and h)
C4	Is (m)	Between (vl and l)	At most (vl)	—	Between (vl and l)
C5	Between (h and vh)	Between (m and h)	Between (l and m)	Between (h and vh)	—

*Pulmonologist*					
C1	—	Between (l and m)	At most (vl)	Between (l and h)	Between (vl and l)
C2	Between (m and h)	—	Between (vl and l)	Is (m)	Between (l and m)
C3	At least (vh)	Between (h and vh)	—	Between (h and vh)	Between (m and h)
C4	Between (l and h)	Is (m)	Between (vl and l)	—	Between (l and m)
C5	Between (h and vh)	Between (m and h)	Between (l and m)	Between (m and h)	—

*Internal medicine physician*					
C1	—	Between (l and m)	Between (vl and m)	Between (m and h)	Between (vl and l)
C2	Between (m and h)	—	Between (l and m)	Is (h)	Is (l)
C3	Between (m and vh)	Between (m and h)	—	Between (h and vh)	Between (vl and m)
C4	Between (l and m)	Is (l)	Between (vl and l)	—	Is (vl)
C5	Between (h and vh)	Is (h)	Between (m and vh)	Is (vh)	—

*Infectious diseases physician*					
C1	—	Between (vl and l)	Between (vl and l)	Between (m and h)	Is (l)
C2	Between (h and vh)	—	Between (m and h)	At least (h)	Between (m and vh)
C3	Between (h and vh)	Between (l and m)	—	Between (h and vh)	Is (h)
C4	Between (l and m)	At most (l)	Between (vl and l)	—	Is (l)
C5	Is (h)	Between (vl and m)	Is (l)	Is (h)	—

**Table 2:** Obtained envelops for the main criteria.

	C1	C2	C3	C4	C5
*Pain physician*					
C1	—	[l, m]	[vl, l]	[h, vh]	[m, h]
C2	[m, h]	—	[l, m]	[vh, vh]	[h, vh]
C3	[h, vh]	[m, h]	—	[vh, ah]	[vh, vh]
C4	[vl, l]	[vl, vl]	[n, vl]	—	[l, m]
C5	[l, m]	[vl, l]	[vl, vl]	[m, h]	—

*Anesthesiologist*					
C1	—	[l, m]	[n, l]	[m, m]	[vl, l]
C2	[m, h]	—	[vl, l]	[h, vh]	[l, m]
C3	[h, ah]	[h, vh]	—	[vh, ah]	[m, h]
C4	[m, m]	[vl, l]	[n, vl]	—	[vl, l]
C5	[h, vh]	[m, h]	[l, m]	[h, vh]	—

*Pulmonologist*					
C1	—	[l, m]	[n, vl]	[l, h]	[vl, l]
C2	[m, h]	—	[vl, l]	[m, m]	[l, m]
C3	[vh, ah]	[h, vh]	—	[h, vh]	[m, h]
C4	[l, h]	[m, m]	[vl, l]	—	[l, m]
C5	[h, vh]	[m, h]	[l, m]	[m, h]	—

*Internal medicine physician*					
C1	—	[l, m]	[vl, m]	[m, h]	[vl, l]
C2	[m, h]	—	[l, m]	[h, h]	[l, l]
C3	[m, vh]	[m, h]	—	[h, vh]	[vl, m]
C4	[l, m]	[l, l]	[vl, l]	—	[vl, vl]
C5	[h, vh]	[h, h]	[m, vh]	[vh, vh]	—

*Infectious diseases physician*					
C1	—	[vl, l]	[vl, l]	[m, h]	[l, l]
C2	[h, vh]	—	[m, h]	[h, ah]	[m, vh]
C3	[h, vh]	[l, m]	—	[h, vh]	[h, h]
C4	[l, m]	[n, l]	[vl, l]	—	[l, l]
C5	[h, h]	[vl, m]	[l, l]	[h, h]	—

**Table 3:** The scale for linguistic terms.

Absolutely low (*n*)	Very low (vl)	Low (l)	Medium (m)	High (h)	Very high (vh)	Absolutely high (ah)
0	1	2	3	4	5	6

**Table 4:** Pessimistic and optimistic preferences for the main criteria.

	C1	C2	C3	C4	C5
*Pessimistic collective preferences*					
C1	—	(vl, 0.2)	(vl, 0.2)	(m, −0.2)	(l, 0.0)
C2	(m, 0.2)	—	(l, −0.2)	(h, 0.0)	(l, 0.0)
C3	(h, 0.0)	(m, −0.0)	—	(h, 0.4)	(m, 0.4)
C4	(l, −0.4)	(l, −0.4)	(vl, 0.2)	—	(vl, 0.4)
C5	(m, 0.4)	(m, −0.2)	(l, −0.4)	(h, −0.2)	—

*Optimistic collective preferences*					
C1	—	(m, −0.4)	(l, −0.2)	(h, 0.0)	(l, −0.4)
C2	(h, 0.2)	—	(l, 0.4)	(vh, −0.4)	(m, 0.4)
C3	(vh, 0.4)	(h, 0.2)	—	(vh, 0.4)	(h, 0.0)
C4	(m, −0.2)	(l, −0.4)	(l, −0.4)	—	(l, 0.0)
C5	(h, 0.4)	(m, 0.2)	(m, 0.4)	(h, 0.4)	—

**Table 5:** Linguistic intervals and utilities for the main criteria.

Criteria	Linguistic intervals	Linguistic utilities	Midpoints	Weights	Rank
C1	[(l, −0.20), (l, 0.50)]	[1.80, 2.50]	2.150	0.147	4
C2	[(m, −0.25), (h, −0.35)]	[2.75, 3.65]	3.200	0.218	3
C3	[(h, −0.30), (vh, −0.25)]	[3.70, 4.75]	4.225	0.288	1
C4	[(vl, 0.45), (l, 0.00)]	[1.45, 2.00]	1.725	0.118	5
C5	[(m, −0.10), (h, −0.15)]	[2.90, 3.85]	3.375	0.230	2

**Table 6:** Weight of the subcriteria.

Criteria		Subcriteria		Weight	Rank
C1	0.147	C11	0.420	0.061	9
		C12	0.374	0.055	10
		C13	0.207	0.030	14

C2	0.218	C21	0.465	0.101	3
		C22	0.224	0.049	12
		C23	0.312	0.068	6

C3	0.288	C31	0.440	0.127	1
		C32	0.343	0.099	4
		C33	0.217	0.062	8

C4	0.118	C41	0.642	0.075	5
		C42	0.358	0.042	13

C5	0.230	C51	0.229	0.053	11
		C52	0.494	0.114	2
		C53	0.276	0.064	7

**Table 7:** The scores for the subcriteria with respect to the alternatives.

Criteria	C1			C2			C3			C4		C5		
Subcriteria	C11	C12	C13	C21	C22	C23	C31	C32	C33	C41	C42	C51	C52	C53
Alt. 1	1	0	0	1	0	0	1	1	1	0	0	1	1	1
Alt. 2	1	0	0	1	0	0	1	0	0	0	0	1	0	1
Alt. 3	1	1	1	0	1	1	0	1	1	1	1	0	0	0
Alt. 4	0	1	1	0	0	0	1	1	1	0	0	1	0	1
*f*_*i*_^*∗*^	1	1	1	1	1	1	1	1	1	1	1	1	1	1
*f*_*i*_^−^	0	0	0	0	0	0	0	0	0	0	0	0	0	0

**Table 8:** Ranking results obtained by weighted VIKOR.

Alternative	*S*_*j*_	Rank	*R*_*j*_	Rank	*Q*_*j*_	Rank
Alt. 1	0, 319	1	0, 075	1	0, 000	1
Alt. 2	0, 594	4	0, 114	2	0, 873	4
Alt. 3	0, 458	2	0, 127	3	0, 752	3
Alt. 4	0, 511	3	0,114	2	0, 721	2

## Data Availability

The data used in this study are available upon request.
